The article "Sustained Exposure to the Widely Used Herbicide Atrazine: Altered Function and Loss of Neurons in Brain Monoamine Systems" was retracted in 2012. Reasons: fabricated or falsified data; an official misconduct investigation; misconduct by an author.

# Sustained Exposure to the Widely Used Herbicide Atrazine: Altered Function and Loss of Neurons in Brain Monoamine Systems

**DOI:** 10.1289/ehp.7783

**Published:** 2005-02-24

**Authors:** Veronica M. Rodriguez, Mona Thiruchelvam, Deborah A. Cory-Slechta

**Affiliations:** Environmental and Occupational Health Sciences Institute, and Department of Environmental and Occupational Medicine, Robert Wood Johnson Medical School, University of Medicine and Dentistry of New Jersey, Piscataway, New Jersey, USA

**Keywords:** atrazine, dopamine, hypothalamus, locomotor activity, microdialysis, prefrontal cortex, striatum, substantia nigra, unbiased stereology

## Abstract

The widespread use of atrazine (ATR) and its persistence in the environment have resulted in documented human exposure. Alterations in hypothalamic catecholamines have been suggested as the mechanistic basis of the toxicity of ATR to hormonal systems in females and the reproductive tract in males. Because multiple catecholamine systems are present in the brain, however, ATR could have far broader effects than are currently understood. Catecholaminergic systems such as the two major long-length dopaminergic tracts of the central nervous system play key roles in mediating a wide array of critical behavioral functions. In this study we examined the hypothesis that ATR would adversely affect these brain dopaminergic systems. Male rats chronically exposed to 5 or 10 mg/kg ATR in the diet for 6 months exhibited persistent hyperactivity and altered behavioral responsivity to amphetamine. Moreover, when measured 2 weeks after the end of exposure, the levels of various monoamines and the numbers of tyrosine hydroxylase-positive (TH^+^) and -negative (TH^−^) cells measured using unbiased stereology were reduced in both dopaminergic tracts. Acute exposures to 100 or 200 mg/kg ATR given intraperitoneally to evaluate potential mechanisms reduced both basal and potassium-evoked striatal dopamine release. Collectively, these studies demonstrate that ATR can produce neurotoxicity in dopaminergic systems that are critical to the mediation of movement as well as cognition and executive function. Therefore, ATR may be an environmental risk factor contributing to dopaminergic system disorders, underscoring the need for further investigation of its mechanism(s) of action and corresponding assessment of its associated human health risks.

Atrazine (ATR; 2-chloro-4-ethylamino-6-isopropylamino-*s*-triazine), a chlorinated member of the family of *s*-substituted triazines, is one of the most widely employed herbicides in the world, with an estimated 76.4 million pounds used annually in the United States alone. It acts to suppress photosynthesis by inhibiting electron transfer at the reducing site of chloroplast complex II (Eldridge et al. 1999). Although it has limited solubility in water, ATR is frequently detected in ground and surface waters in agricultural regions (Colborn and Short 1999). Studies also reveal that ATR can be transported into the home, presumably tracked by soil (Lioy et al. 2000).

Human exposure has been confirmed (Adgate et al. 2001; Clayton et al. 2003), and, in fact, approximately 60% of the U.S. population is exposed to ATR (Birnbaum and Fenton 2003). Recent reports indicate that acute dietary exposures range from 0.234 to 0.857 μg/kg/day, and corresponding figures for chronic dietary exposure are 0.046 to 0.286 μg/kg/day, considering all commodities with U.S. Environmental Protection Agency (EPA) tolerances and drinking water (Gammon et al. 2005). Occupational exposure to ATR, as measured in mixer-loader-tender applicators, was reported to be approximately 2.8 mg ATR/day of work, with an absorbed dose of 1.8–6.1 μg/kg/day based on a 5.6% dermal absorption rate (Gammon et al. 2005). An earlier study of manufacturing workers reported a total ATR exposure of 10–700 μmol (~ 2.157–151.004 mg) per work shift (Catenacci et al. 1993).

The understanding of the potential of ATR to serve as a contributing factor to human disease and dysfunction is currently extremely limited. Epidemiologic studies have linked environmental and/or occupational ATR exposure to increased mortality (Sathiakumar et al. 1996), and to non-Hodgkin’s lymphoma (MacLennan et al. 2003; Sathiakumar and Delzell 1997).

In experimental models, however, a growing experimental literature documents deleterious hormonal and reproductive system effects of ATR. In rodents, reported effects include reductions in testosterone levels; increases in tri-iodothyronine (Friedmann 2002; Stoker et al. 2000, 2002); suppression of immune function (Rooney et al. 2003), of luteinizing hormone (LH), and of prolactin surges (Cooper et al. 2000); the appearance of mammary gland tumors; a disruption of regular ovarian cycles; and the induction of pseudopregnancies (Cooper et al. 1996; Laws et al. 2000).

The effects of ATR on ovarian function in female rats have been ascribed to changes in function of catecholamines in the hypothalamus, specifically decreases in norepinephrine (NE) and increases in dopamine (DA) in this region (Cooper et al. 1998). In correspondence with this observation, *in vitro* studies in PC12 cells show concentration-dependent decreases in intracellular DA after exposure to 12.5–200 μM ATR for 6, 12, 18, and 24 hr and decreases in NE release and intracellular NE concentrations after exposures to 100 and 200 μM ATR for 12, 18, and 24 hr (Das et al. 2000, 2003). In addition, reductions in the expression of DA β-hydroxylase [but not of tyrosine hydroxylase (TH)] were observed. The inhibitory effects of ATR on intracellular NE content and NE release, but not on DA intracellular content, were reversed when PC12 cells were co-incubated with ATR and agents known to enhance transcription, phosphorylation, or activity of TH and DA β-hydroxylase, such as 8-bromo-cAMP, forskolin, or dexamethasone (Das et al. 2003). These findings suggest that ATR could disrupt catecholamine metabolism by altering its biosynthetic enzymes.

The fact that ATR can adversely affect hypothalamic catecholamine systems has notable implications because such effects would be unlikely to be restricted to this particular region, but could affect brain catecholamine systems more generally and thus affect pathways critical to the control of movement (nigrostriatal dopaminergic systems) and of complex cognitive functions (mesocorticolimbic dopaminergic systems). If so, then ATR exposures may also serve as a risk factor for neurodegenerative diseases and/or dysfunctions associated with these systems, which include Parkinson’s disease, schizophrenia, and attention deficit disorder, among others (Crossman 2000; Epstein et al. 1999; Viggiano et al. 2003). Indeed, epidemiologic studies have linked pesticides to an increased odds ratio for Parkinson’s disease (Breysse et al. 2002), and various pesticides that affect catecholaminergic systems have been shown to produce characteristics of Parkinson’s disease in experimental models (Betarbet et al. 2000; Reeves et al. 2003; Thiruchelvam et al. 2000b).

The potential for neurotoxic effects of ATR *in vivo*, however, particularly chronic effects, has received almost no experimental attention. Oral exposure of rats to 1,000 mg/kg ATR for 4–11 days decreased rearing in the open field (Ugazio et al. 1991), whereas acute exposure of rats to 100 mg/kg decreased spontaneous Purkinje cell firing rate and cerebellar potentials evoked by electrical stimulation (Podda et al. 1997).

The objective of the present study was to evaluate the potential for sustained low-level ATR exposure to affect two critical catecholamine pathways of the brain: the nigrostriatal DA pathway, involved in the mediation of movement (Crossman 2000), and the mesocorticolimbic DA pathway critical to complex cognitive functions (Clark et al. 2004; Remy and Samson 2003). For this purpose, we evaluated locomotor activity across the course of exposure, whereas monoamine levels in striatum, prefrontal cortex, nucleus accumbens, and hypothalamus and stereologic cell counts of TH-positive (TH^+^) and TH-negative (TH^−^) cells in the midbrain were evaluated 2 weeks after cessation of exposure. Further, this study sought to determine mechanisms by which any changes in dopaminergic function in these pathways might be produced by examining the acute effects of ATR on striatal DA release using microdialysis.

## Materials and Methods

### Chronic ATR Exposure

#### Subjects, exposure, and experimental design.

Thirty male Long-Evans rats purchased from Taconic Farms (Germantown, NY) were housed individually in plastic cages in a temperature- and humidity-controlled vivarium room with a 12-hr dark/light cycle (lights on 0600 hr). Food intake was restricted to maintain body weights at 300 g, and water was available *ad libitum* during the entire experiment. In our experience, this protocol sustains health and viability to a greater degree than does *ad libitum* feeding. At 9 months of age, exposure to 0, 5, or 10 mg/kg ATR mixed in food was initiated with continuation of *ad libitum* access to distilled drinking water. These doses of ATR were chosen based on reports for the rat of an oral median lethal dose (LD_50_) of 1,869 mg/kg (U.S. EPA 2001), a no observed adverse effect level (NOAEL) of 3.3 mg/kg/day, and a lowest observed adverse effect level (LOAEL) of 34.5 mg/kg/day for this route of administration measured as body weight loss. A chronic dietary NOAEL of 1.8 mg/kg/day and LOAEL of 3.65 mg/kg/day were also reported (U.S. EPA 2001). We recorded body weights and food consumption periodically over the entire duration of the experiment. All procedures were carried out in accord with National Institutes of Health and University of Medicine and Dentistry of New Jersey Animal Use and Care Committee Guidelines (Institute of Laboratory Animal Resources 1996). The experimental design is summarized in Figure 1A.

We recorded locomotor activity at 2, 3, and 6 months of ATR exposure and 2 weeks after cessation of exposure. At the 2-month time point, we measured locomotor activity on 3 consecutive days, with animals receiving an intraperitoneal (ip) injection of saline 5 min before the session during the first 2 days, and an injection of *d*-amphetamine sulfate (1 mg/kg) on day 3. Only a single locomotor activity session was carried out at the 3-and 6-month time points and at 2 weeks after the termination of ATR exposure. Locomotor activity was recorded during the light phase (from 0900 hr to 1300 hr) of the light/dark cycle using methods described below.

Two weeks after cessation of ATR exposure, rats were sacrificed by decapitation, brains were removed, and hypothalamus, prefrontal cortex, nucleus accumbens, and striatum were dissected on ice and frozen for HPLC analysis. The remaining tissue was postfixed in 4% paraformaldehyde for immunohistochemistry and stereologic counts.

#### Locomotor activity measurement.

Each rat was individually placed in an automated locomotor activity chamber equipped with infrared photobeams (Opto-Varimex Minor; Columbus Instruments International Corporation, Columbus, OH). Horizontal, vertical, and ambulatory activities were simultaneously measured and data were collected over the course of a 45-min session.

#### Measurement of monoamine levels.

Tissues were sonicated in 0.1N perchloric acid and centrifuged. Supernatants were stored at −80°C until analyzed for monoamine content. Pellets were digested in 0.5 M sodium hydroxide for measurements of protein concentration using reagents from Bio-Rad (Hercules, CA).

We measured monoamines and their metabolites using HPLC with electrochemical detection as described elsewhere (Thiruchelvam et al. 2000a). Briefly, a Waters pump 515 plus autosampler (Waters Corporation, Milford, MA) was joined to a chromatographic column (Alltech Associates Inc, Deerfield, IL). The amperometric potential was set at 600 mV relative to the silver/silver chloride, and the sensitivity of the detector was set at 100 ρA (microdialysates) or 1 ηA (tissue samples). The mobile phase was an isocratic 0.1 M monobasic phosphate solution containing 0.5 mM sodium octyl sulfate, 0.03 mM EDTA, and 12–14% vol/vol methanol. Results generated by these determinations were analyzed with the Empower Pro program (Empower Software, Waters Corporation) and are expressed in picograms per milliliter of microdialysate or nanograms per milligram of protein of tissue. DA turnover was expressed as the ratio of dihydroxyphenylacetic acid (DOPAC) to DA.

#### Tyrosine hydroxylase immunohistochemistry.

Five randomly selected paraformaldehyde-fixed brains from each treatment group were cut into 30-μm sections, collected in cryoprotectant, and stored at −20°C for immunolabeling studies. Sections were rinsed with 0.1 M phosphate buffer (PB), blocked with 10% normal goat serum for nonspecific binding, and incubated in TH primary antibody (Chemicon, Tamecula, CA) for 48 hr at a dilution of 1:3,500 in PB with 0.3% Triton X-100 and 10% normal goat serum. Sections were then incubated with a secondary antibody 1:200 (Vector Laboratories Inc., Burlingame, CA) overnight. Sections were washed and incubated with avidinbiotin solution from Vectastain ABC reagents (Vector Laboratories) for 1 hr and developed in 3–3′-diaminobenzidine tetrachloride and H_2_O_2_ in 0.05 M Tris buffer. Sections were counterstained with cresyl violet after TH staining. We counted total numbers of TH^+^ and Nissl-stained neurons (TH^−^) in substantia nigra pars compacta (SNpc) and the ventral tegmental area (VTA) using the optical fractionator method as described below.

#### Stereologic analysis.

After delineation of the SNpc and VTA at low magnification (4× objective), one side of every fourth section from the entire midbrain region was sampled at higher magnification (100× objective) using the stereology module of the Stereo Investigator imaging program (MicroBrightField Inc., Williston, VT) with an Olympus Provis microscope (Olympus America, Melville, NY). We used the optical fractionator method, an unbiased quantitative technique, for counting TH^+^ (TH^+^ and cresyl violet^+^ neurons) and TH^−^ (cresyl violet^+^ only) cells. Criteria for TH^+^ and TH^−^ neurons were determined as previously described (Barlow et al. 2004; Thiruchelvam et al. 2004). We determined the mean thickness by measuring two fields from five sections per sample, and the entire depth of field was sampled, ignoring the upper and lower 0.5 μm. All samples were evaluated by one experimenter without knowledge of treatment status.

#### Chemicals.

ATR at 98% purity was purchased from Chem Services Inc. (West Chester, PA). Reagents for microdialysis, HPLC analysis, methylcellulose, and cresyl violet were purchased from Sigma (St. Louis, MO).

### Acute ATR Exposure

#### Subjects, exposure, and experimental design.

Thirty male Long Evans rats weighing between 270 and 320 g purchased from Taconic Farms were habituated to constant standard laboratory conditions of humidity, temperature, and dark/light cycle (lights on 0600 hr) as described above. As shown in Figure 1B, we used microdialysis to evaluate changes in striatal DA release after acute intraperitoneal (ip) exposures to ATR in sessions lasting 7 hr.

#### Surgery.

After a habituation period of at least 1 week, rats were anesthetized with pentobarbital (30–40 mg/kg ip) and every 30 min thereafter received an injection of atropine sulfate (0.3 mg/kg ip) to avoid respiratory failure during the cannula implantation. Once anesthetized (assessed by absence of corneal reflex), the rat was placed in a stereotaxic apparatus (Kopf Instruments, Tujunga, CA), the skull was exposed, and a hole was drilled for placement of a guide cannula (MD-2250; Bioanalytical Systems Inc., West Lafayette, IN) over the right striatum, using stereotaxic coordinates (anterior-posterior, +1.0 mm, medio-lateral, −2.0 mm with reference to bregma, dorso-ventral, −3.4 mm from flat skull) according to the atlas of Paxinos and Watson (1986). The cannula was fixed to the skull with anchor screws and acrylic cement. After surgery, rats were individually housed for a recovery period of 5–7 days with food restricted to keep body weight at 300 g and water was available *ad libitum*.

#### Microdialysis.

A probe of concentric design (MD-2262, tip 2 mm; Bioanalytical Systems, Inc.) was inserted into the guide cannula. The dialysis probe was continuously perfused at a flow rate of 2.5 μL/min through a liquid swivel from an automated system (Bioanalytical Systems Inc.) with a physiologic Ringer’s solution containing 147 mM NaCl, 4.0 mM KCl, 1.2 mM CaCl_2_, and 1 mM MgCl_2_, pH 6.0–6.5. Sample collection occurred every 30 min. The first hour of sampling was discarded to avoid erroneous data due to probe insertion. After three baseline samples, rats received an ip injection of vehicle (1% methyl-cellulose) or ATR (100 or 200 mg/kg), and five subsequent samples of perfusate were collected. In order to probe characteristics of DA release, a high potassium solution (91 mM NaCl, 60 mM KCl, 1.2 mM CaCl_2_, and 1 mM MgCl_2_, pH 6.0–6.5) replaced the normal Ringer’s solution, and two samples were collected under these conditions. Normal Ringer’s solution was subsequently restored, and two additional samples of perfusate were collected. Collection vials contained 3.75 μL 0.1 M HClO_4_ solution. Collected samples were immediately frozen at −80°C until monoamine quantification by HPLC as described above.

#### Histology.

At the completion of micro-dialysis sampling, rats were overdosed with sodium pentobarbital and transcardially perfused with an isotonic saline solution followed by 10% formaldehyde. Brains were postfixed in 10% formalin overnight and then transferred to 30% sucrose. Brains were sectioned in 50 μm coronal slices, mounted, stained with cresyl violet, and coverslipped. Cannula placement for the microdialysis study was confirmed under microscopic analyses.

### Statistical Analyses

We analyzed total locomotor activity counts, body weight, and food consumption using repeated-measures analysis of variance (RMANOVA; treatment × time) followed by post hoc tests as appropriate. Responsivity to *d*-amphetamine and changes in neurotransmitter levels in various brain regions were evaluated by one-way ANOVA with post hoc assessments in the event of main effects of treatment. To provide a more conservative analysis of changes in cell counts, because counts in both regions were derived from the same animals (brains), RMANOVA was carried out based on changes in TH^+^ and TH^−^ cells in both SN and VTA (but not total counts because that was the sum of the TH^+^ and TH^−^ cells), followed by post hoc testing as appropriate. We evaluated the effects of ATR on microdialysis by RMANOVAs with treatment and time as factors, followed by post hoc evaluation in the case of main effects or interactions. In all cases, statistical significance was defined as *p* ≤ 0.05.

## Results

### Chronic ATR Exposure

#### Gross effects of treatment.

No treatment-related changes in body weight or food consumption were detected at any point during the course of the exposure (data not shown), nor did any other signs of overt toxicity manifest at any point.

#### Locomotor activity.

In contrast to the other time points of measurement, the assessment of locomotor activity after 2 months of ATR exposure actually involved three sessions, the first two of which were preceded by an ip injection of saline and the third by 1 mg/kg *d*-amphetamine sulfate. No treatment-related changes in locomotor activity were seen in either of the sessions preceded by saline. However, in the third session, the administration of *d*-amphetamine increased locomotor activity of all three groups relative to levels of activity after saline administration [session 2; *F*(2,26) = 3.63, *p* < 0.041]. Additionally, these increases were modified by ATR treatment in that the 10-mg/kg dose further enhanced locomotor activity by an additional 70% (Figure 2A) relative to the increases in the 0- and 5-mg/kg groups, as confirmed in post hoc analyses.

At the remaining time points of measurement, single locomotor activity sessions were carried out in the absence of drug administration. Under these conditions, after 3 months of ATR exposure, we found pronounced increases in locomotor activity again at the 10-mg/kg dose of ATR [*F*(2,26) = 3.62, *p* = 0.041], with levels of horizontal activity that exceeded those of controls and the 5-mg/kg group by approximately 50% (Figure 2B). These treatment-related effects were also evident in the measurement of locomotor activity at the 6-month time point [*F*(2,24) = 3.45, *p* = 0.048] and again when measured 2 weeks after the termination of ATR treatment [*F*(2,24) = 4.42, *p* = 0.024], when levels remained at 40% above control.

#### Changes in monoamine levels.

Measured 2 weeks after the termination of ATR exposure, changes in DA content (Figure 3A) were significant in striatum [*F*(2,23) = 3.61, *p* = 0.044] as well as in frontal cortex [*F*(2,21) = 3.82, *p* = 0.039]. Statistical analysis confirmed decreased levels of DA (~ 20%) in relation to treatment in striatum, with post hoc assessments indicating efficacy at the 10-mg/kg ATR dose with a similar but nonsignificant trend at 5 mg/kg. In contrast, levels of DA were increased in prefrontal cortex in an inverse U-shaped fashion, with post hoc assessment confirming a significant increase at 5 mg/kg (by 30–40%), with levels declining back toward control values at 10 mg/kg. Both doses of ATR reduced serotonin (5-HT) levels in hypothalamus [Figure 3B; *F*(2,21) = 5.19, *p* = 0.015] by 10–15%. Chronic ATR exposure also decreased levels of NE in frontal cortex [Figure 3C; *F*(2,21) = 3.84, *p* = 0.038], with post hoc assessments showing the effect with the 10-mg/kg dose producing reductions of approximately 15–20%. Although a trend toward increases in NE in nucleus accumbens was suggested, it was associated with significant variability and therefore not statistically significant.

We observed no changes in levels of the metabolites of either 5-HT (5-hydroxyindole acetic acid) or DA [DOPAC, homovanillic acid (HVA)] or DA turnover (DOPAC:DA) in any region.

#### Unbiased stereologic counts of cells in the midbrain.

Changes in numbers of cells in the regions of the cell bodies of the two major DA pathways are shown in Figure 4 for a sample of five randomly selected animals from each treatment group; numbers are shown for TH^+^, TH^−^, and total cells in SNpc and for corresponding data for the VTA. Because these regions were from the same brains, we performed a more conservative statistical analysis based on RMANOVA to examine the impact of treatment on numbers of cells using counts of TH^+^ and TH^−^ from each region (not including total counts). That analysis confirmed a significant main effect of treatment [*F*(2,36) = 5.53, *p* = 0.02] and no interaction of treatment by region, indicating that cell loss occurred in both regions and, moreover, in both TH^+^ and TH^−^ cells. These effects were primarily attributable to the 10-mg/kg dose of ATR, as confirmed in subsequent post hoc tests; the mean reductions in cell numbers ranged from 9 to 13% in the 10-mg/kg dose group, whereas those in the 5-mg/kg group ranged from 0 to 3%.

### Acute ATR Exposure

That systemic administration of ATR can indeed directly affect brain dopaminergic systems was further confirmed in microdialysis experiments. The impact of acute ip administration of ATR (100 or 200 mg/kg) on levels of DA in striatum, as assessed via microdialysis, is presented in Figure 5A. Acutely, ATR significantly decreased basal DA release, as shown in the inset in Figure 5A [main effects: treatment, *F*(2,19) = 4.88, *p* = 0.02; sampling time: *F*(9,18) = 26.77, *p* < 0.0001; treatment by time interaction: *F*(18,171) = 2.77, *p* = 0.0003]. Post hoc tests confirmed decreases as measured at 90, 120, 150, and 180 min postadministration of ATR. By 150 min, the decrements averaged approximately 40% and were seen in both the 100-mg/kg and the 200-mg/kg treatment groups.

We also observed a dose-dependent decrease in DA release when the system was challenged with 60 mM high potassium solution for 60 min [*F*(2,19) = 3.717, *p* = 0.0434]. Although the control group showed a 1,256% increase from baseline in response to potassium (210 min time point), corresponding values for the 100-mg/kg and 200-mg/kg ATR groups were 729 and 427%, respectively, from baseline. After high potassium perfusion, the system was flushed again with normal Ringer’s solution; levels of DA declined in all groups, and no treatment-related differences were evident during the remaining 60 min of sampling. The increase in DA seen in the first sample (240 min time point) after high potassium infusion was due to dead volume of the microdialysis sample collection system.

Analysis of striatal DOPAC levels in the dialysates revealed only a significant effect of sampling time [*F*(9,18) = 13.735, *p* < 0.0001]. One-way ANOVA at each time point did not show any difference among groups in DOPAC concentration during the course of the experiment (Figure 5B). Similarly, analysis of HVA levels showed a significant effect of sampling time [*F*(9,18) = 6.074, *p* < 0.0001] but no effect of group or group × sampling time interaction (Figure 5C).

Administration of vehicle (1% methyl-cellulose) or 100 mg/kg ATR did not result in acute observable effects in these rats, but some rats injected with 200 mg/kg ATR exhibited hypoactivity during the first 2 hr after injection, after which levels appeared normal. Histologic analysis confirmed that cannula placement was appropriately located in dorsal striatum for all rats.

## Discussion

The present study demonstrates that sustained low-level ATR exposure in diet can adversely affect both major long-length dopaminergic tracts of the central nervous system, resulting in persistent increases in locomotor activity, alterations in responsivity to the indirect DA agonist amphetamine, changes in monoamine levels, and, ultimately, loss of neurons in the midbrain. Thus, adverse effects of ATR are not restricted to endocrine and reproductive systems or to hypothalamic regions of brain. The effects observed here cannot be ascribed to acute toxicity because the half-life of ATR in tissue ranges from 31.3 to 38.6 hr, and 95% of the ATR administered is excreted within 7 days of dosing, whereas changes in monoamines and numbers of neurons were measured 2 weeks posttreatment. Moreover, the doses used here did not produce any changes in body weight or food consumption or any signs of overt toxicity.

The observations of protracted changes in neurotransmitter levels coupled with neuronal loss have particular significance, given the critical roles of the nigrostriatal and mesocorticolimbic dopaminergic systems in controlling fine motor behavior and complex cognitive function, respectively (Clark et al. 2004; Crossman 2000; Remy and Samson 2003). Dysfunctions of dopaminergic systems include Parkinson’s disease, schizophrenia, attention deficit disorder, and learning and memory impairments. Collectively, the present findings raise the possibility that ATR exposure could be a contributory risk factor for such disorders.

Chronic ATR exposure caused cell loss not only to TH^+^ immunoreactive cells but also to TH^−^ cells in the VTA and SNpc. The non-dopaminergic neuronal subpopulation in these regions includes GABAergic (Deniau et al. 1978), calbindin (Gerfen et al. 1985), and cholecystokinin-like immunoreactive neurons (Seroogy and Fallon 1989). The lack of selectivity of effects makes it likely that ATR will exhibit neurotoxicity, including cytotoxicity to other neuronal populations in other brain regions, although other regions were not examined in the present study. Additionally, ATR may exert neurotoxic effects on other cell types of the brain as well, such as glial cells. The specificity and mechanism(s) of ATR effects within the central nervous system remain to be determined, and such assessments are clearly warranted based on the findings presented here.

Chronic ATR increased locomotor activity, an effect present after 3 months of exposure, persisted for 6 months and was still evident even 2 weeks after cessation of exposure. Moreover, rats treated for 2 months with 10 mg/kg ATR exhibited an enhanced locomotor activity response to a *d*-amphetamine challenge. Amphetamine is known to promote the release of DA and a decrease in its re-uptake into the presynaptic terminal (Cooper et al. 2003). Thus, the increases in locomotor activity could reflect ATR-induced up-regulation of striatal DA receptors, as might be expected to occur in response to the corresponding reduction in basal DA levels (Figure 3A) or DA release produced by ATR (Figure 5A). Placement in a novel environment such as the locomotor activity chamber could increase DA, activating up-regulated DA receptors and thereby producing hyperactivity (Badiani et al. 1998), a hypothesis in agreement with the increases in locomotor activity induced by amphetamine sulfate (Mao et al. 2001).

The locomotor hyperactivity observed here differs from findings of a previous study in which 1,000 mg/kg ATR administered for 4–11 days decreased rearing in the open field (Ugazio et al. 1991). Such decreases could reflect acute toxicity of a high dose of ATR because the chemical was administered immediately before the behavioral evaluation in that study, coupled with a decline in DA release that would accompany its administration and be expected to reduce activity levels, as was observed.

The reductions noted here in levels of DA, NE, and 5-HT observed, respectively, in striatum, prefrontal cortex, and hypothalamus at the 10-mg/kg ATR dose could be due to inhibitory effects on synthesis in these monoamine pathways. Precursors of DA and NE (tyrosine) and of 5-HT (tryptophan) undergo the same hydroxylation process via TH or tryptophan hydroxylase, respectively. Both enzymes are pteridin-dependent aromatic amino acid hydroxylases and are highly homologous, reflecting a common evolutionary origin from a single genetic locus (Cooper et al. 2003). In an *in vitro* study using PC12 cells in which NE and DA were decreased by ATR, the NE effect was reversed when cells were co-incubated with agents known to enhance transcription and phosphorylation of dopamine β-hydroxylase and TH (Das et al. 2003), consistent with the possibility that ATR may have inhibitory effects on these enzymes.

Previous studies have reported changes in hypothalamic DA and/or NE levels after acute ATR administration at 100 mg/kg by gavage to male rats (Cooper et al. 1998). We did not observe such changes in the chronic exposure paradigm used here, a difference that could reflect initiation of compensatory mechanisms to maintain a constant production of these neurotransmitters under conditions of chronic exposure. Alternatively, catecholamine levels were determined in specific hypothalamic nuclei in that study, whereas here we examined the hypothalamus in its entirety, thus possibly diluting any regional changes (Cooper et al. 1998).

Chronic ATR exposure did decrease hypothalamic 5-HT levels, effects consistent with its known alterations of neuroendocrine systems, including the release of LH and prolactin. Serotonergic neurons from the dorsal and medial raphe nuclei project to hypothalamus, activating the hypothalamo–pituitary–adenocortical (HPA) and the hypothalamo–pituitary–gonadal (HPG) axes in the rat (Fuller 1996; Jorgensen et al. 1998). Agents that disrupt 5-HT transmission are known to alter the HPA and HPG axes (Fuller 1996; Fuller and Snoddy 1990). Furthermore, selective degeneration of the midbrain dorsal and ventromedial region of the hypothalamus induced by 5,7-dihydroxytryptamine reduces LH levels (van de Kar et al. 1980). Taken together, it can be inferred that reductions in hypothalamic 5-HT resulting from ATR could affect both the HPA and HPG axes and thereby alter other organ systems of the body with which these systems interact.

DA and NE alterations in prefrontal cortex are also notable given the critical role of this structure in mediating executive function, including working memory (Dreher et al. 2002). Dysfunction of this region is also involved in cognitive deficits, altered stress responsivity, hyperactivity disorder, and schizophrenia (Mostofsky et al. 2002; Tam and Roth 1997; Viggiano et al. 2003). An increase in cortical DA levels, such as observed at 5 mg/kg, could be due to an increase in DA synthesis, decreased degradation, or altered re-uptake. It is worth noting that autoreceptors on DA terminals in the prefrontal cortex regulate release but not synthesis of DA (Cooper et al. 2003), which may explain why augmented DA concentrations in this region are not corrected after ATR exposure.

Findings from the microdialysis component of these experiments are consistent with such an assertion and show alterations in the dynamics of DA in striatum after acute ATR treatment. A dose-dependent decrease in striatal DA release as observed here would normally trigger compensatory mechanisms such as decreased re-uptake rate and increased production and release of DA. As is evident from Figure 5, none of these compensatory mechanisms appears to be operative, at least within the time frame encompassed by these experiments.

The observed decline in both basal and stimulated DA release could have several explanations. First, it could reflect a generalized inhibition of DA synthesis, given the absence of group differences at the end of the experiment. DA is distributed mainly in two functional presynaptic compartments, a cytoplasmic pool and a vesicular pool. Potassium-induced release is Ca^2+^ dependent and occurs from the vesicular pool (Du et al. 1999), which is the newly synthesized pool (Lamensdorf et al. 1996). Another possibility is that ATR decreases the firing rate of striatal and/or SN neurons, decreasing DA release. Additionally, TH exists in two kinetic forms, with differential affinities for tetrahydrobiopterin (cofactor for TH). The proportion of TH in the high-affinity state appears to be a function of neuronal firing rate (Cooper et al. 2003). A dose of 100 mg/kg ATR decreased cerebellar cell firing rate after 60 and 90 min, with rates returning to normal by 180 min; this inhibitory effect lasted up to 180 min after exposure to 200 mg/kg ATR (Podda et al. 1997). ATR could also be acting on ionotropic GABA receptors. Binding of RO15-4513 (an inverse agonist of the GABA_A_ receptor benzodiazepine site) was inhibited when cortical membranes were incubated with ATR (Shafer et al. 1999). This would increase the influx of chloride ions, leading to hyperpolarization of cells, preventing depolarization that would, in turn, decrease DA release.

No changes in levels of the DA metabolites DOPAC and HVA were observed in the microdialysis component of this study, although DA levels were altered. DA is converted to DOPAC intraneuronally after re-uptake, whereas extraneuronal DA is converted to HVA by the enzymes catechol-*O*-methyltransferase and monoamine oxidase. The lack of change in DOPAC and HVA could reflect the relatively modest nature of the changes in DA, leaving a sufficiently high concentration of DA in the intracellular space to maintain constant levels of DOPAC and HVA production. Further, DA re-uptake was not impaired. The decreases in DOPAC and reductions in extracellular DOPAC and HVA after potassium stimulation across sampling time in the microdialysis component of this study agree with results of other such studies (Holson et al. 1998; Robinson and Camp 1991; Stanford et al. 2000; Westerink and Tuinte 1986) and may reflect initial damage caused by the probe insertion, which recovers after several hours. The decrease in DOPAC levels that occurs with the increase in extracellular DA after potassium perfusion is thought to reflect a decrease in intracellular DA metabolism by monoamine oxidase (Camarero et al. 2002).

At the present time, the health-related impacts that ATR exposures may exert in human populations remain unknown. Assessments of occupational exposures have been limited, and systematic studies of environmental exposures have not been undertaken. Although the doses of ATR used in these studies are higher than those estimated for human exposures, additional considerations must be applied to such comparisons. First, data projecting human exposure are always limited because they are dependent upon when exposures occurred relative to the time of measurement and do not provide measurement of the tissue of interest (i.e., the brain) in such cases. Second, the doses used here are low for the experimental species (rat), being consistent with previously reported NOAEL and LOAEL levels. Furthermore, even at these levels, the doses may not have been as high as administered because probably not all the ATR ingested would have been absorbed; a portion of it could have been easily eliminated through the feces, suggesting that lower actually absorbed doses could underlie the deleterious effects observed in this study.

In summary, the collective findings from this study demonstrate that ATR may have broad effects on brain monoamine systems and thereby influence a wide range of behavioral functions. Clearly, additional studies are needed to unravel the targets of ATR and the mechanism(s) of its effects, as well as the ultimate human health consequences of such exposures for behavioral and/or neurologic dysfunctions.

## Figures and Tables

**Figure 1:** Experimental designs for the chronic ATR exposure component of the study (*A*) and for acute ATR exposure for microdialysis studies (*B*). Abbreviations: MC, methylcellulose; SNpc, substantia nigra pars compacta.

**Figure 2:** Horizontal locomotor activity (group mean as percentage of control ± SEM). (*A*) Effect of a 1-mg/kg dose of amphetamine sulfate administration on locomotor activity after 2 months of ATR exposure. (*B*) Spontaneous locomotor activity measured at 3 months and 6 months of ATR exposure, and 2 weeks after cessation of ATR exposure. RMANOVA was followed by Fisher’s post hoc test. Absolute values (total counts ± SEM) for control animals are 8094.44 ± 1822.95 (amphetamine sulfate challenge after 2 months of ATR exposure); 3860.56 ± 703.66 (3 months of ATR exposure); 3168.60 ± 550.36 (6 months of ATR exposure), and 4257.00 ± 588.45 (2 weeks after cessation of ATR). TX, treatment.
*Significantly different from control group, *p* < 0.05 (*n* = 8–10 rats per treatment group).

**Figure 3:** Levels of DA (*A*), 5-HT (*B*), and NE (*C*; presented as the group mean as a percentage of control ± SEM) in striatum, prefrontal cortex, nucleus accumbens, and hypothalamus 2 weeks after cessation of ATR exposure (6 months). One-way ANOVAs for each region were followed by Fisher’s post hoc test. Absolute values (ng/mg protein ± SEM) for control animals are, for DA: 122.25 ± 8.54 (striatum), 2.83 ± 0.21 (prefrontal cortex), 6.09 ± 0.55 (hypothalamus), 78.70 ± 7.12 (nucleus accumbens); for 5-HT: 2.46 ± 0.27 (striatum), 15.45 ± 1.31 (prefrontal cortex), 14.44 ± 0.46 (hypothalamus), 8.22 ± 0.68 (nucleus accumbens); and for NE: 11.44 ± 0.77 (prefrontal cortex), 34.65 ± 1.67 (hypothalamus), 1.63 ± 0.14 (nucleus accumbens).
*Significantly different from control group, *p* < 0.05 (*n* = 7–10 rats per treatment group).

**Figure 4:** Numbers of TH^+^, TH^−^, or total cells in SNpc (top row) or in VTA (bottom row) measured using unbiased stereology and determined 2 weeks after termination of ATR treatment. Each point represents the value for an individual animal, with *n* = 5 randomly selected per treatment group counted. Black bars represent group medians.

**Figure 5:** Time course (group mean as percentage of basal release ± SEM) of striatal release of DA (*A*; baseline DA release shown in inset), DOPAC (*B*), and HVA (*C*) over the course of microdialysis. Microdialysates were collected every 30 min; high potassium infusion (60 mM K^+^) lasted 1 hr, after which normal Ringer’s solution was restored for 1 hr longer. The presence of response in the first sample after high potassium was due to the dead volume of the microdialysis sample collection system. +100-mg and *200-mg groups significantly different from control group, *p* < 0.05 (*n* = 7–8 rats per treatment group).
